# Relationship between Financial Asset Allocation, Leverage Ratio, and Risk-Taking of Small- and Medium-Sized Enterprises in China: Taking Environment-Related Industries as an Example

**DOI:** 10.1155/2022/2431428

**Published:** 2022-06-13

**Authors:** Qing Chen

**Affiliations:** School of Economics and Management, Yiwu Industrial and Commercial College, Yiwu 322000, China

## Abstract

With the improvement of environmental policies and industry requirements for enterprise production and management, small- and medium-sized enterprises in environment-related industries were also changing. It was known from the existing research that the investment allocation of assets of small- and medium-sized enterprises was closely related to risk and return, and the leverage ratio of enterprises affected the risk-taking level of enterprises. In the process of sustainable development, enterprises will inevitably bear certain risks, but excessive risk-taking will bring all kinds of uncertainty and bankruptcy risk to the expected income and future cash flow of enterprises. Therefore, taking small- and medium-sized enterprises in environment-related industries as an example, this paper put forward relevant assumptions by analyzing the interaction between the existing enterprise financial asset allocation, risk-taking level and leverage ratio. In order to facilitate empirical analysis, A-share listed companies in environment-related industries in Shanghai and Shenzhen stock exchanges, small- and medium-sized board and GEM listed companies in Shenzhen stock exchange from 2007 to 2019 were selected as research samples. These data came from the information open platform for small- and medium-sized enterprises in environment-related industries, the research reports of third-party consulting companies and CSMAR and Wind databases. The empirical results showed that the allocation of financial assets had a significant impact on the level of risk-taking, and there was a *U*-shaped relationship between them when other conditions remained unchanged. At the same time, the financial asset allocation of small- and medium-sized enterprises in Chinese environment-related industries had a significant impact on the enterprise leverage ratio. Under other conditions unchanged, there was a *U*-shaped relationship between the two. In addition, leverage played an intermediary role in the relationship between financial asset allocation and risk-taking level. In addition to directly affecting the allocation of financial assets, it can also indirectly affect the risk-taking level of enterprises through leverage ratio.

## 1. Introduction

As an important part of the Chinese economy, small- and medium-sized enterprises play an important role in increasing government revenue and national income, stabilizing employment, and stimulating economic vitality. However, due to the reallocation of resources, the competition between related industries and the lack of government supervision over enterprises, some small- and medium-sized enterprises discharge pollutants at will, which has brought certain harm to the surrounding and world environment, resulting in social criticism of enterprises related to the environmental industry [1]. At present, Chinese economic development has entered a new normal. Under the influence of macro policies and cyclical fluctuations, enterprises related to the environmental industry are affected by factors such as rising raw material prices and increasing labor costs. The development of the main business of most enterprises slows down or even stagnates, and the profits deviate from the balance of supply and demand. With the increasing requirements of countries around the world for enterprises related to the environmental industry, the risk-taking level of small- and medium-sized enterprises related to the environmental industry continues to decline, and the survival time and survival rate of small- and medium-sized enterprises continue to decline. Therefore, the risk control and undertaking of nonfinancial enterprises have attracted much attention. On the contrary, the profit margin of the financial market represented by stocks and funds is much higher than the average profit margin of the real estate industry [2]. Therefore, in order to pursue a higher return on investment, the operators of small- and medium-sized enterprises related to the environmental industry began to allocate financial assets, from traditional stocks, bonds, funds to credit loans, purchase financial products, invest in financial institutions, and so on. Enterprise financial investment has become a hot trend, and small- and medium-sized enterprises are no exception. At the same time, Chinese small- and medium-sized enterprises related to the environmental industry have been facing the problem of high enterprise leverage [3]. The so-called enterprise leverage refers to the use of debt and a small amount of capital to leverage a large number of assets, so as to expand production and investment activities. From the relationship between the company's capital structure and the company's leverage ratio which is actually the asset liability ratio, which can be expressed by the ratio of total liabilities to total assets. It reflects the conflict of interest and optimal adjustment between shareholders and creditors and affects the normal sustainable operation of the enterprise to a certain extent. The change of asset investment allocation increases the uncertainty of investment income, and the change of enterprise leverage ratio will inevitably affect the risk-taking level of enterprises.

Through the data investigation and comparative study of enterprises in environment-related industries, such as textile and real estate, it is found that among the enterprises that choose to invest in financial products, some enterprises optimize the investment structure and increase the company's profits by allocating financial assets [4]. However, in the face of the temptation of a high-yield virtual economy, some nonfinancial enterprises invest in high-risk and high-yield financial assets, resulting in the deterioration of their financial situation. Therefore, the problem of how financial asset investment affects enterprise leverage and risk-taking has attracted the extensive attention of relevant scholars at home and abroad. Although risk-taking is an inevitable requirement for enterprises to obtain profits and returns, too high enterprise risk-taking will also increase the overvaluation of their expected income, increase the uncertainty of long-term cash flow. And expose them to bankruptcy risk. Therefore, taking enterprises in environment-related industries as an example, this paper successively analyzed various factors that may affect the development of small- and medium-sized enterprises, such as financial asset allocation, enterprise leverage, and risk-taking level, and put forward relevant assumptions on this basis. Through the research on the relationship between financial asset allocation, enterprise leverage, and risk-taking level of small- and medium-sized enterprises, this paper used empirical analysis to explore the main factors affecting the development of enterprises related to environmental industry.

## 2. Related Works

For enterprises in environment-related industries, the change of enterprise leverage ratio is usually reflected in the dynamic adjustment process of the enterprise capital structure. The earliest research comes from the theory of enterprise capital structure, which mainly studies the financing behavior of enterprises. For the long-term and high-quality development of enterprises, financing is essential, and there have been early capital structure theory, modern capital structure theory, new capital structure theory, and related applications. In the monitoring of the enterprise leverage ratio, some scholars evaluate the enterprise leverage ratio through the ratio between total liabilities and total assets from a micro perspective, or use the asset liability ratio to measure the enterprise leverage ratio [5]. Others use the ratio between short-term corporate liabilities and current assets to represent the enterprise leverage ratio, or use the ratio between the current loan amount and the total assets at the beginning of the period to calculate the enterprise leverage ratio. Other scholars use the ratio of short-term liabilities to total assets to measure the leverage ratio of enterprises.

Some scholars have studied the influencing factors of enterprise risk-taking related to environmental industries from the aspects of monetary policy and the nature of enterprise ownership. Some people have studied environment-related small- and medium-sized enterprises from the perspective of the impact of monetary policy, and found that there is a positive correlation between enterprise leverage and risk-taking, while monetary policy has an asymmetry on enterprise risk-taking, which can jointly affect enterprise risk-taking [6]. With the tightening of the national monetary policy, the risk bearing capacity of enterprises will be reduced, and there will be asymmetric effects between different enterprises and industries to a certain extent. For example, monetary policy has a transmission effect on enterprise risk assessment and management and is affected by certain economic cycle fluctuations. The rise of interest rates caused by monetary policy is easy to promote the increase of high-risk loans and debt risk. In addition, in view of the relationship between the nature of ownership and enterprise risk-taking, some scholars have found that the risk-taking degree of non-state-owned enterprises is lower than that of state-owned holding enterprises, and the enterprise risk-taking degree presents an inverted *U*-shaped relationship with the separation of control and management rights [7]. Compared with non-state-owned enterprises, state-owned small- and medium-sized enterprises have a more effective inhibitory effect on the level of risk-taking.

In recent years, some people have explored the impact of corporate management and board governance in environment-related industries on corporate risk-taking. The research shows that the enterprise management shareholding higher than the threshold will increase the enterprise risk-taking level. The relationship between professional managers and enterprise risk-taking is related to the incentive level of enterprises. Giving managers a certain proportion of equity can reduce the company's risk, while the management shareholding of the enterprise is too high or too low, and the risk bearing level is very high [8]. After managers get an equity incentive, they will improve the company's performance and increase the company's risk-taking, and then the stock price will rise. With the increase of managers' shareholding, in order to pursue a high return, they are more inclined to invest in high-risk projects. The manager's shareholding will make him averse to high-risk, so the risk-taking level of the company will be reduced. After empirical analysis of multinational data, some scholars found that there is a positive correlation between enterprise risk-taking and the degree of state protection of its investors. The share transfer right will increase the company's risk-taking, and the shareholding level and scale of the board of directors are negatively correlated with the company's risk-taking. There is a significant positive correlation between the number of independent directors and the shareholding ratio of the board of directors and corporate risk-taking [9]. Generally, there is a positive correlation between the number of shareholders and the level of risk-taking, and there is a positive correlation between the independence of the board of directors and the risk-taking of the company. Private equity ownership has a positive impact on the company's risk-taking. Some scholars have found that there is a significant negative correlation between agency cost and risk-taking. In addition, there is a positive correlation between managers' overconfidence and enterprise risk-taking.

## 3. Related Theories and Research Hypothesis Design

### 3.1. Correlation Theory

#### 3.1.1. The Relationship between Financial Asset Allocation and Enterprise Risk-Taking

In view of the relationship between enterprise performance and enterprise risk-taking in environment-related fields, generally, enterprises with a high risk-taking level are often accompanied by large capital investment expenditure, which is also the key to the normal operation and development of enterprises. Research shows that companies with a high risk-taking level usually have higher *R* & *D* investment and innovation enthusiasm, and the company is more competitive [10]. Risk-taking by enterprises can help enterprises grow and improve corporate performance, and risk can also significantly enhance corporate value to a certain extent. Generally, there is a *U*-shaped, inverted *U*-shaped or positive correlation between enterprise performance and risk-taking; that is, the higher the level of risk-taking, the higher the enterprise value and capital allocation efficiency.

Due to the particularity of environment-related industries, for the relationship between executive compensation and enterprise risk-taking in environment-related fields, executive compensation incentives may be negatively correlated with enterprise risk-taking. Previous studies have shown that the stock option incentives of enterprise executives in environment-related fields will increase corporate risk, and there is a positive correlation between executive compensation, stock price sensitivity, and return volatility [11]. Therefore, increasing executive compensation can inhibit the negative impact of free cash flow on enterprise risk-taking. There is a positive correlation between enterprise risk-taking and executive compensation in environment-related fields, a negative correlation with enterprise scale, a negative correlation with equity concentration, a positive correlation with the shareholding ratio of management, and a significant positive correlation with the asset liability ratio of the company.

Affected by the limited resources of environmental industries, enterprises need to make full use of scarce resources to maximize profits and need to coordinate and reasonably allocate among major industries and financial assets. Therefore, the allocation of financial assets is to meet the basic asset allocation requirements of not putting eggs in the same basket. From the research on the impact of financial asset allocation on relevant factors of enterprises, it is known that financial asset allocation may increase the risk bearing of enterprises to a certain extent, which is not conducive to the long-term development of enterprises [12]. For example, financial asset investment not only has a significant negative effect on the investment rate of enterprises in environment-related fields, but also the degree of financial investment is directly related to the level of risk-taking. However, because the allocation of financial assets can play the role of “reservoir” to a certain extent, it can appropriately reduce the risk of enterprises. Some scholars have found that the allocation of financial assets can adjust the cyclical fluctuation of enterprise income, make the asset structure more reasonable, and reduce the financing risk of enterprises [13]. Relevant studies have shown that financial asset investment can inhibit enterprises' risk-taking to a certain extent, but driven by dividends in the Chinese financial market, enterprises usually increase their investment in risky financial assets under the influence of short-term high returns. Because the enterprise's capital is fixed, the allocation of financial assets may affect the enterprise's risk-taking. The allocation of financial assets will inevitably reduce the working capital in the enterprise budget, which will affect the uncertainty of operating income and the risk bearing of the enterprise.

#### 3.1.2. The Relationship between Financial Asset Allocation and Corporate Leverage Ratio

According to existing research, the influencing factors of enterprise leverage in environment-related industries mainly include macro and micro levels. From the macro level, the overall economic prosperity and recession affect the credit level, thus affecting the leverage ratio of enterprises. Improving the capital utilization ratio can reduce the debt ratio of enterprises. The nature of enterprises is different, and their sensitivity to macroeconomic changes is also different, resulting in different levels of leverage. Different levels of leverage lead to different sensitivity to the macro economy. In different stages of economic development, the leverage ratio shows different trends at the micro and macro levels [14]. Therefore, economic expectations are different, and the state's control of leverage is also different. From the micro perspective, the impact of leverage mainly includes the change of debt ratio, the adjustment direction of industrial structure, productivity, and inflation. The CEO has a great influence on the leverage ratio of the company. Payable income tax and individual income tax have a certain impact on enterprise leverage. Through the research of dynamic panel data and system generalized moment model, some scholars know that financial investment can reduce the leverage ratio of listed companies, but it is not suitable for nonlisted companies. The adoption of financial financing by enterprises often leads to excessive dependence on high leverage, aggravating the actual capital structure and deviating from the goal. At the same time, leverage has a certain impact on enterprises, the economy, and finance. For the impact of leverage on enterprise management performance, the company's leverage ratio has a significant negative correlation with operating performance, which means that reducing leverage ratio can help to improve operating performance, and appropriate liabilities can promote the company's operating performance. For the impact of leverage on enterprise investment, the high leverage of enterprises has seriously inhibited enterprise investment, so it must be deleveraged. In addition, leverage also has a certain impact on the economy and finance [15]. For example, there is usually an upper limit on corporate debt. Exceeding this limit will hinder the improvement of enterprise productivity and inhibit economic growth when corporate debt exceeds 90%. At the same time, a too high leverage ratio will also expand the impact on the financial system and reduce financial stability.

Similar to the relationship between financial asset allocation and enterprise risk-taking level, according to the existing research, the relationship between financial asset allocation and enterprise leverage is mainly reflected in two aspects: (1) financial asset allocation inhibits the rise of enterprise leverage. The increase in the share of financial assets will inhibit the leverage ratio of enterprises. The share of financial assets plays the role of “reservoir,” which is an effective way for small- and medium-sized enterprises to deal with the shortage of funds and solve the urgent need [16]. There is a significant negative correlation between the share of financial assets, the profitability of financial channels, and the leverage ratio of enterprises, and the allocation of financial assets is expected to prevent risks. There is a nonlinear relationship between overall financial investment and enterprise leverage. The leverage ratio at both ends of the financial asset allocation structure is higher than that in the middle region. The level of financial investment can inhibit financial risks. At present, the financial leverage of listed nonfinancial enterprises in China is inversely proportional to the degree of financial investment. (2) The allocation of financial assets intensifies the financial risk of enterprises and improves the leverage ratio of enterprises. Under the downward pressure of the economy, the profitability of entity enterprises related to the environmental industry continued to decline due to the impact of macro policies and cyclical fluctuations. However, financial asset dividends stimulate the financial asset allocation of small- and medium-sized enterprises [17]. Entrepreneurs' profit-seeking psychology enables them to increase debt financing and increase enterprise leverage to obtain high profits and returns. The improvement of the profitability of financial channels has significantly improved the leverage ratio of enterprises. Special attention should be paid to the risk of enterprises relying too much on financial investment profits. The research data show that the allocation of financial resources is unreasonable. Enterprises with low asset turnover and a growth rate of small- and medium-sized enterprises have more financial asset allocation, which leads to a sharp rise in the overall leverage ratio of enterprises [18]. Excessive debt and sustained negative profits will increase the role of financial asset allocation in improving leverage and weaken the inhibition of leverage.

#### 3.1.3. The Relationship between Corporate Leverage Ratio and Risk-Taking

At present, the relationship between leverage ratio and risk-taking level is mostly studied from the perspective of the banking industry. Generally speaking, the capital level is inversely proportional to the bank's risk-taking ability. As a policy management tool, the leverage ratio plays an important role in reducing bank financial risks [19]. The enterprise leverage ratio, that is, the enterprise asset liability ratio, is the ratio of enterprise debt financing to total assets. It measures the financial risk level of enterprises to a certain extent. Through borrowing, enterprises can alleviate the shortage of funds required for investment. The uncertainty of investment is the premise for enterprises to improve their risk-taking level. It is known from the existing research results that through enterprise deleveraging, the risk-taking ability of enterprises can be significantly improved, which has a far greater impact on small- and medium-sized enterprises than on large enterprises. The capital structure of listed enterprises in environment-related industries has a significant positive impact on the level of risk-taking. The higher the asset liability ratio, the lower the risk bearing level of the enterprise. Short-term debt helps to improve the risk-taking level of enterprises, and the deleveraging of nonfinancial enterprises has a *U*-shaped relationship with risk-taking. Deleveraging of companies with a high asset liability ratio will reduce their risk-taking, while deleveraging of companies with less debt will increase their risk-taking [20]. In highly leveraged companies, entrepreneurs prefer high-risk projects to a certain extent. They will also choose high-yield and high-risk projects by borrowing funds, so as to increase the risk-taking of enterprises. From the above research on the relationship between financial asset allocation and enterprise risk-taking, enterprise leverage, and enterprise investment in financial assets, it is known that although financial asset allocation bears the risks brought by financial asset allocation, it also enjoys the benefits brought by financial asset allocation. Financial investment can weaken financial risk-taking by reducing leverage.

### 3.2. Research Hypothesis Design and Empirical Route

From the research results of small- and medium-sized enterprises in environment-related industries in terms of financial asset allocation, risk-taking ability, and leverage ratio, it is known that there is a certain internal relationship between them. In order to further explore the correlation between them, this paper puts forward the following research hypotheses:

**Hypothesis 1 .**

The allocation of corporate financial assets has a significant impact on the level of risk-taking, and when other conditions remain unchanged, there is a *U*-shaped relationship between the two.

**Hypothesis 2 .**

The financial asset allocation of enterprises has a significant impact on the leverage ratio of enterprises. And when other conditions remain unchanged, there is a *U*-shaped relationship between the two.

**Hypothesis 3 .**

Corporate leverage ratio plays a mediating role in the impact of financial asset allocation on the level of corporate risk-taking.

In order to test the above research hypotheses, this paper designs the following research route for empirical analysis and evaluates the relevant propositions, as shown in Figure 1.

## 4. Relevant Index Definition and Model Construction

### 4.1. Relevant Index Definition

#### 4.1.1. Explained Variable

Enterprise risk-taking (Risk) is mainly measured by the volatility of corporate earnings, the annual volatility of stock returns, the maximum and minimum difference in return on assets, the possibility of enterprise survival, and tolerance for corporate failure. For comprehensive consideration, this paper uses the standard deviation of return on assets (*ROA*) in the three-year rolling window period to measure the volatility of enterprise income. In order to avoid the interference of industry heterogeneity on the results, it is necessary to adjust the *ROA* of each enterprise to the industry average *ROA*, that is, the enterprise *ROA* minus the industry average *ROA* to obtain the adjusted return on assets (*adjROA*). Finally, the enterprise risk-taking index is obtained by calculating the standard deviation of *adjROA* in the three-year rolling window period. The calculation formula is as follows:

(1) $$\begin{array}{c} {\text{Risk}}_{i,t}=\sqrt{\frac{1}{T-1}\sum_{t=1}^{T}{\left(\text{adj}ROA_{i,t}-\frac{1}{T}\sum_{t=1}^{T}\text{adj}ROA_{i,t}\right)}^{2}}, \end{array}$$

where *T* is the rolling window length, *i* represents the specific *i* th enterprise, and *t* denotes the number of year during the observation period, its value range is 1–3.

#### 4.1.2. Explanatory Variable

Financial asset investment of enterprises is expressed in *fin*. The proportion of the sum of financial monetary funds, trading financial assets, financial derivatives, available for sale financial assets, held to maturity investment, entrusted loans and financial products, and long-term equity investment in the total assets of the enterprise is taken as the proxy variable of the enterprise's financial investment behavior. The larger the index, the greater the proportion of investment in financial assets.

#### 4.1.3. Mediating Variable

As an intermediary variable, enterprise leverage ratio (*Lev*) is mainly measured by asset liability ratio, and its value can be expressed as total liabilities/total assets.

#### 4.1.4. Control Variable

It is known from the existing research that the following indicators can usually be used as control variables: enterprise size (*Size*), operation period (*Age*), growth capacity (*Growth*), and initial profitability (*ROA*). In order to describe the macro level, the following indicators can be used as control variables: GDP growth rate (*GDP*), social financing scale growth rate (*Social*), annual dummy variable (*Year*), and industry dummy variable (*IND*).

The specific variable definitions are shown in Table 1.

### 4.2. Model Construction

Because there is a certain internal relationship between the enterprise's risk-taking model and the enterprise's leverage ratio; that is, the current situation is affected by the previous results, and the expected dynamic panel deviation, growth ability, and profitability make the control variables such as sales growth rate prone to endogenous problems. Therefore, based on existing research, this paper uses the system generalized moment estimation model (GMM) to study the relationship between financial asset allocation, leverage ratio, and risk-taking of small- and medium-sized enterprises [21].

In order to verify the correctness of hypothesis 1, combined with relevant data analysis, the regression method can be used to test the relationship between financial asset allocation and the risk-taking level of small- and medium-sized enterprises. The model is as follows:

(2) $$\begin{array}{c} {\text{Risk}}_{i,t}=\alpha_{0}+\alpha_{1}{\text{Risk}}_{i,t-1}+\alpha_{2}{\text{Fin}}_{i,t}+\sum \alpha_{i}Z_{i,t}+\varepsilon_{i,t}, \end{array}$$

(3) $$\begin{array}{c} {\text{Risk}}_{i,t}=\beta_{0}+\beta_{1}{\text{Risk}}_{i,t-1}+\beta_{2}{\text{Fin}}_{i,t}^{2}+\beta_{3}{\text{Fin}}_{i,t}+\sum \beta_{i}Z_{i,t}+\varepsilon_{i,t}. \end{array}$$

If hypothesis 1 is true, that is, when other conditions remain unchanged, the financial asset allocation of small- and medium-sized enterprises is positively correlated with the level of risk-taking, then the coefficient *β*_2_ of Fin_*i*,*t*_^2^ should be positive.

Similarly, in order to prove the correctness of hypothesis 2, this paper uses the following model to test the relationship between financial asset allocation and enterprise leverage:

(4) $$\begin{array}{c} {\text{Lev}}_{i,t}=\gamma_{0}+\gamma_{1}{\text{Lev}}_{i,t-1}+\gamma_{2}{\text{Fin}}_{i,t}+\sum \gamma_{i}Z_{i,t}+\varepsilon_{i,t}, \end{array}$$

(5) $$\begin{array}{c} {\text{Lev}}_{i,t}=\delta_{0}+\delta_{1}{\text{Lev}}_{i,t-1}+\delta_{2}{\text{Fin}}_{i,t}^{2}+\delta_{3}{\text{Fin}}_{i,t}+\sum \delta_{i}Z_{i,t}+\varepsilon_{i,t}. \end{array}$$

If hypothesis 2 is true, that is, under other conditions unchanged, the financial asset allocation of small- and medium-sized enterprises is positively correlated with the enterprise leverage ratio, then the coefficient *δ*_2_ of Fin_*i*,*t*_^2^ should be positive.

In order to prove the correctness of hypothesis 3, this paper uses the following model to test the mediation effect:

(6) $$\begin{array}{c} Y=cX+\varepsilon_{1},\\ M=aX+\varepsilon_{2},\\ Y=c^{\prime }X+bM+\varepsilon_{3}, \end{array}$$

where *X*, *M*, and *Y* represent three different variables respectively. *c* is the total effect of *X* on *Y*, *a* is the effect of *X* on *M*, *b* is the effect of *M* on *Y*, *ab* is the intermediate effect, and *c*′ is the direct effect. The relationship between the effect coefficients is: *c*=*c*′+*ab*.

In order to describe the intermediary effect of leverage, this paper uses the intermediary effect model to study the relationship between different variables. The model is as follows:

(7) $$\begin{array}{c} {\text{Risk}}_{i,t}=\theta_{0}+\theta_{1}{\text{Risk}}_{i,t-1}+\theta_{2}{\text{Fin}}_{i,t}+\theta_{3}{\text{Lev}}_{i,t}+\sum \theta_{i}Z_{i,t}+\varepsilon_{i,t}. \end{array}$$

According to models (1), (3), and (5), the intermediary effect of leverage ratio needs to meet the following conditions: (1) Enterprise risk-taking and financial asset allocation are regressed, and the regression coefficient *α*_2_ reaches a significant level. (2) The enterprise leverage ratio and financial asset allocation are regressed, and the regression coefficient *γ*_2_ is significant. (3) The level of enterprise risk-taking regresses simultaneously with the financial asset investment and leverage ratio, and the coefficient of the intermediate variable *θ*_3_ is significant. When the coefficient of financial asset investment *θ*_2_ is not significant, the leverage ratio exerts a full mediation effect. When *θ*_2_ is significant, the leverage ratio exerts a partial mediation effect.

## 5. Demonstration and Analysis

### 5.1. Sample Selection

This study selects A-share listed companies in Shanghai and Shenzhen stock markets, small- and medium-sized boards, and GEM listed companies in the Shenzhen Stock Exchange from 2007 to 2019 as research samples.  Figure 2 shows the annual distribution of IPO of sample enterprises in environment-related industries. These data mainly come from the information open platform for small- and medium-sized enterprises in environment-related industries, the research reports of third-party consulting companies, and CSMAR and Wind databases. The macro data for GDP and CPI come from the National Bureau of Statistics, the Ministry of Finance, the People's Bank of China and other departments. The selected data does not include large enterprises, financial and real estate companies, ST or PT companies, samples with incomplete data and missing data for three consecutive years, and companies with significant financial anomalies. Finally, STATA 16.0 and SPSS 22.0 are used to process the characteristic data of small- and medium-sized enterprises in environment-related industries while avoiding the interference of outliers.

### 5.2. Data Description and Statistics

The descriptive statistics of the main variables are shown in Table 2. It can be seen from Table 2 that the standard deviation of the enterprise risk-taking level (*Risk*) is 1.9062, the minimum value is 0.0020, and the maximum value is 95.6825, which shows that the risk-taking levels of different companies in different years are obviously different. The maximum value of financial asset allocation is 0.5012, and the minimum value is 0.0000. From the proportion of the financial asset allocation of a single enterprise in the finance of the whole enterprise, we can know that there are great differences in the financial asset allocation of enterprises in different years. The average leverage ratio of enterprises is 0.4526, and the maximum value is 0.9422, which reflects that the leverage ratio of Chinese enterprises is too high, and there are great differences among different enterprises related to the environmental industry.

For each explanatory variable in Table 1, we adopt the Pearson correlation coefficient test. The testing results are shown in Table 3. According to the statistical results, the correlation coefficient between most explanatory variables is small, indicating that there is no deep multicollinearity between explanatory variables. Therefore, the multiple regression method can be used to further analyze the relationship between them. Therefore, it can be determined that the model settings are correct. The correlation coefficient between financial asset allocation, leverage ratio, and enterprise risk-taking is small and positive, indicating that there is a positive correlation between them and there is not much linear correlation. This indicates that there may be a nonlinear relationship between them, which verifies the hypothesis of a nonlinear relationship between variables in hypothesis 1 and hypothesis 2, but the exact relationship needs to be further verified by the regression results. The analysis of the correlation coefficient of each variable shows that the variance expansion factor is far less than the threshold of 10, which further explains the rationality of the model.

In addition, we can get the change trend of risk-taking level and leverage ratio of sample enterprises in environment-related industries in the five years before and after IPO from 2008 to 2018, as shown in Figure 3. Among them, the risk-taking level shows an increasing trend, while the change in leverage ratio is relatively stable.

### 5.3. Regression Result Analysis

The specific regression results of the dynamic panel systematic generalized method of moments are shown in Tables 4 and 5. GMM estimation has a one-step method and a two-step method. The two-step method has parameters and excessive dependence on the standard deviation, so the results are biased downward and inaccurate. Although the one-step estimation method has low regression efficiency, it can ensure the consistency of estimation. Therefore, the one-step method is mostly used in practical applications.

The empirical results show that the change of enterprise risk-taking level (*L*. *Risk*) lagging for a period is significantly positively correlated with the current risk-taking level, which reflects the stickiness of the risk-taking level of small- and medium-sized enterprises related to the environmental industry in China.

By comparing the regression results and hypotheses, we find that the square coefficient (*Fin*^*2*^) of financial asset allocation in model (3) is 0.4513, which is significantly positive at the level of 1%. It confirms the research hypothesis H1: the allocation of corporate financial assets has a significant impact on the level of risk-taking, and when other conditions remain unchanged, there is a *U*-shaped relationship between the two. According to the parameter estimation results of model (5), the square coefficient (Lev^2^) of the enterprise leverage ratio is significantly positive at the level of 1%, which supports the research hypothesis 2. The financial asset allocation of enterprises has a significant impact on the leverage ratio of enterprises. And when other conditions remain unchanged, there is a *U*-shaped relationship between the two. In model (7), the coefficients of financial asset allocation share (Fin) and corporate leverage ratio (Lev) are both significantly positive at the level of 5%, which confirms hypothesis 3. It illustrates that corporate leverage ratio plays a mediating role in the impact of financial asset allocation on the level of corporate risk-taking. Financial asset allocation not only exerts direct influence on enterprise risk-taking but also exerts indirect influence through the adjustment of the leverage ratio.

### 5.4. Robustness Test

In order to test the robustness of the above regression results, by changing the calculation method of risk, this paper uses the difference between the maximum and minimum of the three-year rolling window length of the environmental industry adjusted return on assets (adj*ROA*) to measure the enterprise's risk-taking level, which is recorded as Risk_2_. The results obtained by regression estimation are shown in Table 5. It can be seen from Table 5 that the test and analysis results obtained by using the model constructed in this paper are basically consistent, which reflects that the established model has good robustness.

In addition, the Sobel test and the Bootstrap method are used to test the robustness of the intermediary effect of the company's leverage ratio. The regression estimation results are shown in Table 6. When taking risk-taking as the explanatory variable, the *Z* value of the Sobel test is significantly positive, which confirms the significant existence of an intermediary effect, accounting for 53.62%. In the test results using the Bootstrap method, the confidence interval of the indirect effect does not include 0, so the intermediary effect is significant. Therefore, by changing the measurement method of the explained variable, Risk_2_ is basically consistent with the previous risk estimation, indicating that the model has good robustness.

## 6. Conclusion

Affected by various factors, such as environmental policies and industry requirements for enterprise development, the allocation of financial assets of small- and medium-sized enterprises related to environmental industry in China had a significant impact on the level of risk-taking. Under other conditions unchanged, there was a *U*-shaped relationship between them. When the allocation ratio of financial assets was in the middle position, it mainly acted as a reservoir and restricted the risk-taking to a certain extent. However, if the ratio is too low or too high, giving up profits and speculative profits will increase the risk-taking level of enterprises. At the same time, the financial asset allocation of small- and medium-sized enterprises related to the Chinese environmental industry had a significant impact on the enterprise leverage ratio. Under other conditions unchanged, there was a *U*-shaped relationship between the two. Leverage ratio in an appropriate range was conducive to inhibit the risk-taking of enterprises, and too low or too high leverage ratio will promote the risk-taking of enterprises. In addition, the leverage ratio played an intermediary role in the relationship between the degree of financial investment and the level of risk-taking. In addition to the direct impact of financial asset allocation, it can also indirectly affect the risk-taking level of enterprises through leverage ratio. Through the empirical research on the financial asset allocation, enterprise leverage and risk-taking of enterprises related to environmental industry, this paper put forward the following suggestions: (1) Enterprises should reasonably allocate financial assets. Make use of the role of financial assets in solving the cash flow of enterprises and make the allocation of financial assets play the role of reservoir and risk prevention savings by increasing liquidity, so as to resist the fluctuations of macro policies and economic cycles. (2) Establish an enterprise risk control and early warning mechanism to maintain the enterprise leverage at a reasonable level and avoid relying on debt financing. (3) Government departments should continue to promote the smooth progress of supply side structural reform, prevent the hollowing out of assets, broaden enterprise financing channels, establish and improve the risk monitoring of enterprise departments under the national system, and remind enterprises to pay attention to the risks brought by macro policies and economic cycle fluctuations.

## Figures and Tables

**Figure 1:** Schematic diagram of relevant proposition design and empirical test scheme.

**Figure 2:** Annual distribution of IPO of sample enterprises in environment-related industries.

**Figure 3:** Change trend of risk-taking level and leverage ratio of sample enterprises in environment-related industries in the five years before and after IPO.

**Table 1:** Variable definition, symbols, and descriptions.

Variable definition	Variable name	Symbol	Definition
Explained variable	Enterprise risk-taking	*Risk*	Standard deviation of three-year rolling enterprise return on assets
Mediating variable	Leverage ratio	*Lev*	Gross liabilities/total assets

Explanatory variable	Financial assets investment	*Fin*	The proportion of the sum of the trading financial assets seven items in the balance sheet to the total assets of the enterprise
	Enterprise scale	*Size*	Natural logarithm in total assets
	Operating years	*Age*	Natural logarithm of years of establishment plus 1
	Growth ability	*Growth*	Revenue growth rate
	Initial profitability	*ROA*	The earnings before interest and tax/total assets

Control variable	GDP growth	*Gdp*	GDP growth
	Growth in the scale of social financing	*Social*	Growth in the scale of social financing
	Industry	*IND*	Industry dummy variable
	Annual	*Year*	Annual dummy variable

**Table 2:** Descriptive statistics of main variables.

Variable	Observed value	Mean	Standard deviation	Minimum value	Maximum value
*Risk*	38522	1.8533	1.9062	0.0020	95.6825
*Lev*	33195	0.4526	0.1988	0.0493	0.9422
*Fin*	33195	0.0497	0.0875	0.0000	0.4873
*Size*	36512	25.6994	0.7062	21.6354	28.6231
*Age*	39536	13.5326	6.2282	2.0000	32.0000
*Growth*	31562	0.1953	0.4169	-0.3864	2.1478
*ROA*	36512	9.6846	8.9695	-14.9156	44.6982
*Gdp*	37892	8.6167	2.1326	6.6000	14.2000
*Social*	37892	15.6895	30.6523	-13.9654	98.8864

**Table 3:** The Pearson correlation coefficient matrix of the variable.

	*Risk*	*Lev*	*Fin* ^*2*^	*Fin*	*Size*	*Age*	*Growth*	*Roa*	*Gdp*	*Social*
*Risk*	1.000									
*Lev*	0.033^*∗∗∗*^	1.000								
*Fin* ^*2*^	0.236^*∗∗∗*^	−0.023^*∗∗*^	1.000							
*Fin*	0.227^*∗∗∗*^	−0.016^*∗∗*^	0.956^*∗∗∗*^	1.000						
*Size*	−0.036^*∗∗∗*^	0.195^*∗∗∗*^	0.031^*∗∗∗*^	0.297^*∗∗∗*^	1.000					
*Age*	−0.008^*∗*^	0.264^*∗∗∗*^	0.226^*∗∗∗*^	0.037^*∗∗∗*^	0.315^*∗∗∗*^	1.000				
*Growth*	−0.013^*∗*^	−0.075^*∗∗∗*^	−0.069^*∗∗∗*^	0.028^*∗∗∗*^	−0.019^*∗∗∗*^	0.320^*∗∗∗*^	1.000			
*Roa*	0.026^*∗∗∗*^	−0.162^*∗∗∗*^	−0.153^*∗∗∗*^	−0.306^*∗∗*^	−0.362^*∗∗∗*^	−0.019^*∗∗∗*^	−0.096^*∗∗∗*^	1.000		
*Gdp*	0.029^*∗∗∗*^	−0.019^*∗∗*^	−0.014^*∗∗*^	0.135^*∗∗∗*^	−0.226^*∗∗∗*^	−0.356^*∗∗∗*^	0.068^*∗∗∗*^	0.165^*∗∗∗*^	1.000	
*Social*	0.021^*∗∗∗*^	−0.003	−0.002	0.086^*∗∗∗*^	−0.126^*∗∗∗*^	−0.235^*∗∗∗*^	−0.010^*∗*^	−0.095^*∗∗∗*^	0.365^*∗∗∗*^	1.000

*Notes*. ^*∗*^, ^*∗∗*^, ^*∗∗∗*^ mean significant at the level of 10%, 5% and 1% respectively.

**Table 4:** The estimation results of system GMM.

Variable	*Risk*	*Risk*	*Lev*	*Lev*	*Risk*
	Model (2)	Model (3)	Model (4)	Model (5)	Model (7)
L.lev			0.8236^*∗∗∗*^ (0.012)	0.8137^*∗∗∗*^ (0.014)	
*L.Risk*	0.1384^*∗∗∗*^ (0.043)	0.1431^*∗∗∗*^ (0.041)			0.1265^*∗∗∗*^ (0.040)
*Lev*					0.0832^*∗∗*^ (0.036)
*Fin*	0.2746^*∗∗*^ (0.126)		0.1062^*∗∗∗*^ (0.034)		0.1894^*∗∗*^ (0.095)
*Fin* ^*2*^		0.4513^*∗∗∗*^ (0.134)			
*Lev* ^*2*^				0.7956^*∗∗∗*^ (0.023)	
*Size*	−0.1186^*∗∗∗*^ (0.139)	−0.1231^*∗∗∗*^ (0.167)	−0.0265^*∗∗∗*^ (0.093)	−0.0289^*∗∗∗*^ (0.101)	0.1102^*∗∗*^ (0.046)
*Age*	0.0162^*∗∗*^ (0.007)	0.0234^*∗∗*^ (0.011)	0.0017^*∗∗*^ (0.001)	0.0019^*∗∗*^ (0.003)	0.0134^*∗∗*^ (0.006)
*Growth*	0.1326^*∗∗*^ (0.062)	0.1452^*∗∗*^ (0.049)	0.0058^*∗∗∗*^ (0.007)	0.0062^*∗∗∗*^ (0.009)	0.1107^*∗∗*^ (0.052)
*Roa*	−0.0029 (0.002)	−0.0042 (0.003)	−0.00036^*∗∗∗*^ (0.000)	−0.00039^*∗∗∗*^ (0.001)	−0.0025 (0.002)
*Gdp*	0.0186^*∗∗∗*^ (0.006)	0.0192^*∗∗∗*^ (0.011)	−0.0042^*∗∗∗*^ (0.001)	−0.0046^*∗∗∗*^ (0.002)	0.0203^*∗∗∗*^ (0.007)
*Social*	0.0006^*∗∗∗*^ (0.000)	0.0009^*∗∗∗*^ (0.000)	0.0001^*∗∗*^ (0.000)	0.0003^*∗∗*^ (0.000)	0.0006^*∗∗∗*^ (0.000)
Constant term	2.2286^*∗∗∗*^ (0.796)	3.1256^*∗∗∗*^ (0.8023)	0.6439^*∗∗∗*^ (0.089)	0.7726^*∗∗∗*^ (0.093)	1.9011^*∗∗∗*^ (0.650)

*Notes*. Standard error in parentheses; ^*∗*^, ^*∗∗*^, ^*∗∗∗*^ mean significant at the level of 10%, 5%, and 1%, respectively.

**Table 5:** Robustness test to change the estimation method of risk-taking.

Variable	*Risk2*	*Risk2*	*Lev*	*Lev*	*Risk2*
	Model (2)	Model (3)	Model (4)	Model (5)	Model (7)
L. lev			0.8236^*∗∗∗*^ (0.012)	0.8137^*∗∗∗*^ (0.014)	
*L. Risk*	0.1384^*∗∗∗*^ (0.043)	0.1431^*∗∗∗*^ (0.041)			0.1289^*∗∗∗*^ (0.040)
*Lev*					0.0816^*∗∗*^ (0.036)
*Fin*	0.2746^*∗∗*^ (0.126)		0.1062^*∗∗∗*^ (0.034)		0.2136^*∗∗*^ (0.095)
*Fin* ^*2*^		0.4513^*∗∗∗*^ (0.134)			
*Lev* ^*2*^				0.7956^*∗∗∗*^ (0.023)	
*Size*	−0.1186^*∗∗∗*^ (0.139)	−0.1231^*∗∗∗*^ (0.167)	−0.0265^*∗∗∗*^ (0.093)	−0.0289^*∗∗∗*^ (0.101)	−0.1023^*∗∗*^ (0.046)
*Age*	0.0162^*∗∗*^ (0.007)	0.0234^*∗∗*^ (0.011)	0.0017^*∗∗*^ (0.001)	0.0019^*∗∗*^ (0.003)	0.0022^*∗∗*^ (0.006)
*Growth*	0.1326^*∗∗*^ (0.062)	0.1452^*∗∗*^ (0.049)	0.0058^*∗∗∗*^ (0.007)	0.0062^*∗∗∗*^ (0.009)	0.0996^*∗∗*^ (0.052)
*Roa*	−0.0029 (0.002)	−0.0042 (0.003)	−0.00036^*∗∗∗*^ (0.000)	−0.00039^*∗∗∗*^ (0.001)	−0.0023^*∗∗∗*^ (0.002)
*Gdp*	0.0186^*∗∗∗*^ (0.006)	0.0192^*∗∗∗*^ (0.011)	−0.0042^*∗∗∗*^ (0.001)	−0.0046^*∗∗∗*^ (0.002)	0.0189^*∗∗∗*^ (0.007)
*Social*	0.0006^*∗∗∗*^ (0.000)	0.0009^*∗∗∗*^ (0.000)	0.0001^*∗∗*^ (0.000)	0.0003^*∗∗*^ (0.000)	0.0006^*∗∗∗*^ (0.000)
Constant term	2.2286^*∗∗∗*^ (0.796)	3.1256^*∗∗∗*^ (0.8023)	0.6439^*∗∗∗*^ (0.089)	0.7726^*∗∗∗*^ (0.093)	1.8865^*∗∗∗*^ (0.695)

*Notes*. Standard error in parentheses; ^*∗*^, ^*∗∗*^, ^*∗∗∗*^ mean significant at the level of 10%, 5%, and 1%, respectively.

**Table 6:** Robustness test of mediating effect of leverage ratio.

Dependent variable	Sobel test value		Bootstrap (95%) confidence interval	
	*Z* value	The effect proportion (%)	Upper limit	Lower limit
Risk	5.866^*∗∗∗*^	53.62	0.0012	0.0233
Risk_2_	5.838^*∗∗∗*^	61.23	0.0015	0.0245

*Notes*. ^*∗∗∗*^ mean significant at the level of 1%.

## Data Availability

The labeled dataset used to support the findings of this study is available from the corresponding author upon request.
